# Integrated Analysis of lncRNA-miRNA-mRNA ceRNA Network in Mixed Dry Eye Disease

**DOI:** 10.1155/2022/1534142

**Published:** 2022-05-17

**Authors:** Zhongxia Tang, Yu Zhang, Haoyang Wu, Chunhua Liu, Yunyu Lian, Haocong Ling, Xiang Li, Xiaohe Lu

**Affiliations:** ^1^Department of Ophthalmology, Zhujiang Hospital, Southern Medical University, Guangzhou, China; ^2^The Second School of Clinical Medicine, Zhujiang Hospital, Southern Medical University, Guangzhou, China; ^3^Department of Ophthalmology, Shenzhen Hospital, University of Chinese Academy of Sciences, Shenzhen, China; ^4^Shenzhen Key Laboratory of Viral Vectors for Biomedicine, Shenzhen Institutes of Advanced Technology, Chinese Academy of Sciences, Shenzhen, China

## Abstract

In order to investigate the relationship between inflammation and lncRNA in mixed dry eye disease (DED), this study establishes competitive endogenous RNA (ceRNA) network in mixed DED. Microarray analysis of cornea from mixed DED mice is performed to screen for differences in lncRNA and target genes, and miRNA bioinformatics were predicted based on the ceRNA hypothesis. The ceRNA network, which consists of 96 relationship pairs, is constructed using the top 10 upregulated lncRNAs and all upregulated mRNAs and two pairs of lncRNA-miRNA-mRNA pairs (NONMMUT047964.2-miR-671-5p-Egr-1andNONMMUT054540.2-miR-1934-5p-Grm2) are selected for RT-qRCR verification in mouse corneal epithelial cells under high osmotic pressure and the samples for microarray. Meanwhile, mouse corneal epithelial cell lines (MCECs), transfected siRNA of NONMMUT047964.2 under high osmotic pressure, shows a decrease in apoptosis rate and a decrease in expression of IL-1*β* and IL-6. The experimental results show that the NONMMUT047964.2-miR-671-5p-Egr-1 axis may regulate the inflammation and promote the apoptosis of corneal epithelial cells under hypertonic condition.

## 1. Introduction

Dry eye is a common multifactorial disease of the ocular surface, which Asian race is a significant risk factor [1]. Meanwhile, this disease prevalence, range from 5 to 50%, has increased significantly with the growth in screen time on computers and mobile phones and the general use of masks during the Covid-19 pandemic. TFOS DEWS II report identified the two primary categories of dry eye as evaporative and aqueous deficient, although they had potential overlap [2].The core mechanism of dry eye disease (DED) is tear hyperosmolarity which activating MAPK signaling pathways leads to the release of inflammatory mediators and proteases [3].These inflammatory factors and hyperosmolarity will lead to characteristic punctate epithelial injury and tear film instability, in some cases will form a vicious circle to aggravate ocular surface injury and determines the chronicization of the process, with damage of the nerve fibers. The cornea is the densest part of the body's nervous system, and inflammatory factors make the nerves more sensitive to corneal damage. To date, the management of chronic ocular pain remains a real therapeutic challenge in Ophthalmology. Patients with neuropathic pain are often advised to take long term steroids, but there also bring risk of ocular hypertension, cataracts and opportunistic infections [4]. Nerve Regenerative Therapy and systemic administration of anticonvulsants, tricyclic antidepressants (e.g., Nortriptyline) have begun to be used clinically, but sometimes still not provide adequate relief from pain [5].

Long non-coding RNAs (lncRNAs), non-coding RNAs that are more than 200 nucleotides, can regulate a variety of biological processes, including epigenetic modification, variable RNA splicing, and protein stability. There is growing evidence that lncRNAs play significant roles in the biological processes of neuroinflammation, neuropathic pain, and eye disease. miRNAs are small endogenous non-coding RNAs that are found to be differentially expressed in DED [6]. Salmenal et al. proposed the hypothesis of competitive endogenous RNA (ceRNA), which revealed that lncRNAs can act as competing endogenous RNAs (ceRNAs) to alter target genes expression by competitively binding to the miRNA binding site. In the last few years, lncRNAs have gradually demonstrated its great research value in ophthalmic diseases. For example, the lncRNAs TUG1 (taurine upregulated gene 1) is found to promote the progress of murine retina differentiation [7]. LncRNAs MIAT alleviates corneal angiogenesis by promoting proliferation and migration of human umbilical vein endothelial cells. The ceRNA networks connected to lncRNA have been shown to play a significant role in a range of inflammatory disorders. However, no ceRNA network of hybrid dry eye has been constructed. Consequently, it is essential to investigate the role of ceRNA networks in hybrid dry eye. We may be able to gain insight into the pathogenesis of dry eye and find a link between the onset of DED and neuroinflammation, which may lead to solutions to the most pressing challenges of chronic pain caused by dry eye.

In the current study, we analyze the expression profile of lncRNAs in a mouse model of mixed DED using the microarray analysis. In our findings, several significantly altered lncRNAs, rarely studied, have been found. Then, a ceRNA network, which contained 7 lncRNAs, 23 miRNAs, and 58 mRNAs, is constructed for the first time. Meanwhile, NONMMUT047964.2 is found as a potential risk element of lncRNAs involved in the inflammation of DED through miR-671-5p/Egr-1 axis, implying a novel target for early therapy.

### 1.1. Related Work

Dry eye disease, a common, accompanied by inflammation and pain, is often classified as evaporative dry eye and aqueous deficient dry eye, mixed dry eye, and so on. As the epidemic spread across the globe, the use of face masks increased dramatically. The use of a mask causes the exhaled air to flow upward, passing through the eye surface and promoting evaporation of water from the eye surface, increasing the risk of dry eye. Long-term use of mobile phones or computers, staring at the screen for too long may lead to reduced tear secretion, increases the risk of dry eye disease water shortage. The overlap of risk factors of evaporative dry eye and water-deficient dry eye makes the study of mixed dry eye more clinically significant, but the studies on mixed dry eye are no enough. Long non-coding RNA (lncRNA) is usually involved directly or indirectly in various biological processes and signaling pathways, and its powerful multi-functional regulatory network may be associated with some symptoms of dry eye [8,9]. In addition, the role of lncRNA in the pathogenesis and treatment of ocular diseases such as Glaucoma and Cataract have been well established, but the mechanisms involved in dry eye disease have not been fully elucidated. The inflammation and neuropathic pain of dry eye has been of concern. The neuroactive ligand-receptor interaction signaling pathway activated by lncRNA increases the level of 5-hydroxytryptamine in the tear, which mediates ocular surface inflammation by increasing the tear 5-hydroxytryptamine [10]. Meanwhile, lncRNAs have been shown to be associated with neuropathic pain, and a number of different expression lncRNAs have been identified in pain-related areas of the mouse, rat, and human nervous systems, such as the dorsal root ganglia and spinal cord. In addition, it has been suggested that lncRNAs contribute to the development and maintenance of neuropathic pain by modulating pain-related genes and increasing neuronal excitability in the primary sensory neurons of the dorsal Root Ganglia [11,12]. The pathogenesis of DED is complex, heterogeneous, and is still not fully elucidated. At the same time, in the face of inflammation and neuropathic pain caused by dry eye, there is still a lack of reliable therapeutic targets. In order to better understand the abnormal gene expression regulation of mixed DED and look for possible therapeutic targets, we first simulated tear-deficiency dry eye with subcutaneous injection of scopolamine and exposed to a dry and flowing environment to simulate evaporative dry eye disease, so as to construct a mixed dry eye disease mouse model. Then the differentially expressed endogenous RNA is confirmed in this model via microarray analysis and a ceRNA network is constructed through multiple screening and verification.

The present study also predicted that the NONMMUT047964.2 may be involved in dry eye disease through the miR-671-5p/Egr-1 axis by regulating the inflammatory signal pathway in MCECs. In the previous studies, miR-671-5p has often been shown to exhibit anti-inflammatory effects. Inhibited miR-671-5p in orbital fat stem cells would result in release macrophage pro-inflammatory cytokine [13,14]. miR-671-5p has been found to reduce the inflammation of human rheumatoid arthritis fibroblast-like synoviocytes by inhibiting the expression of STAT3. Xi et al. found that overexpression of miR-671-5P could reduce chondrocyte apoptosis and inflammatory injury. Early Growth Response-1(Egr-1) has been shown to play an important role in inflammatory processes in various tissues. For example, inflammation is promoted in animal models of cholestatic liver injury, ischemia reperfusion lung injury, and arteriosclerosis formation with the increase of Egr-1 expression level. It has been shown that Egr-1, when combined with the DNA sequence of the promoter region, can activate a variety of downstream target genes, including microsomal Prostaglandin *e* synthase-1(mPGES-1), which binds to cyclooxygenase 2(COX-2) to produce PGE2, suggested that Egr-1 is involved in the induction of prostaglandins [15–17]. Upregulation of NONMMUT047964.2,Egr-1 and downregulation of miR-671-5p is observed in cornea of mixed DED mice and MCECs under hypertonic conditions. After transfection with siRNA of NONMMUT047964.2, MCECs also showed downregulation of Egr-1 and upregulation of miR-671-5p, suggesting that NONMMUT047964.2 may promote the expression of inflammatory factor (IL-1*β* and IL-6) and apoptosis of MCECs through miR-671-5p/Egr-1 axis. However, the specific mechanism still needs to be further studied, and more convincing experiments are needed to illustrate this conclusion, which is also the focus of our team's future research.

There still have several limitations to the study. First, we have only preliminarily verified the relationship between some ceRNA pairs at the mRNA level, but we lack more sufficient experimental evidence to prove the direct relationship between lncRNA, miRNA, and mRNA. Second, we only preliminarily verified that NONMMUT047964.2 can reduce the inflammatory level of MCECs, but the more specific mechanism has not been studied. Besides, we did not knock down lncRNA in the DED animal model to observe whether the corneal epithelial injury of DED mice can be reversed and whether the level of inflammation can be reduced. This will be the future research direction of our team.

## 2. DE Mouse Model and Corneal Fluorescein Sodium Staining Score

### 2.1. DE Mouse Model

Fifty specific-pathogen-free (SPF) female C57BL/6J mice (100 eyes), 8 weeks old, weighing 18–20.5 g, obtained from the breeding facility of Zhuhai Pepsistone Biotechnology Co., Ltd, are randomized into two groups (control group *n* = 25, DE group *n* = 25). DE and control group are housed in an environmentally controlled room (25°C and 12 h/12 h light–dark cycle), with adequate rodent chow food and water available. The only difference is that DED mice are in a 30% humidity environment, which maintained continuous air flow, and 60% humidity in the rooms of controls. DE and control groups are pharmacologically induced by the subcutaneous injection of 0.5 mg/0.2 mL scopolamine hydrobromide or 0.2 mL normal saline, respectively, at 8 a.m., 12 noon, 4 p.m. and 8 p.m. daily. Schirmer's I-test and the corneal fluorescein sodium staining score are recorded before and at days 14, 28 after treatment. Each mice is anesthetized by intraperitoneal injection of tribromine ethanolamine (1.25 g/ml).

### 2.2. Detection of Basal Tear Secretion

The tear secretion quantity is examined by Schirmer's I-test at 0, 2, and 4 weeks after starting the experiment, which is one of the important indexes in the diagnosis of dry eye. After intraperitoneal injected tribromine ethanolamine (0.2 ml/10 g) to anesthetize, cotton thread (Tianjin Jingming New Technological Development Co., Ltd) is placed at the vault about one-third of the distance from the outer corner of the mouse's lower eyelid and gently close the mouse's eyelids for 30 seconds. The length (mm) of the wet cotton thread is measured and recorded.

### 2.3. Corneal Fluorescein Sodium Staining Score

After anesthetizing mice by intraperitoneal injecting tribromine ethanolamine (0.2 ml/10g), 1% fluorescein sodium solution (Tianjin Jingming New Technological Development Co., Ltd) is dropped into the conjunctival sac of each eye and the score is then evaluated with cobalt-blue light under a slit lamp microscope by an experienced oculist. Since pigmentation of the cornea indicates that the corneal epithelium is damaged, we set up a scoring system. Cornea, divided into four quadrants, is checked and recorded the scores independently, 0 points indicates non-pigmentation of the corneal epithelium; 1 point indicates that the pigmented area exists but fewer than 30 dots; 2 points represent that pigmented area accounts more than 30 but not diffuse; 3 points suggest that the pigmented area diffuse but not patchy and 4 points indicate that fluorescent plaques have formed. The final score is obtained by adding the scores of each quadrant of the cornea of the same mouse, ranging from 0 to 16 points.

### 2.4. Corneal Morphology and Epithelial Thickness

The eyes are removed and fixed in eyeball fixed liquid and embedded in paraffin. The eyes are sectioned at a thickness of 4 μ m in the vertical plane. The sections passing through the optic disc are stained with hematoxylin and eosin (H&E). All slides are digitally scanned at 20x resolution using 3D HISTECH Pannoramic MIDI (Budapest, Hungary) and the corneal epithelium thickness of the central area are evaluated on digitalized pictures using the 3D HISTECH software CaseViewer (version 2.3.0) by one masked observer.

### 2.5. Microarray Analysis

Agilent Mouse ceRNA Microarray 2019 (4∗180K, Design ID:086242) is used in this study and data analyses of the 6 RNA samples is extracted from DED mouse cornea which are performed by OE Biotechnology Co., Ltd., (Shanghai, China). The lncRNAs are identified by the Noncode database (http://www.noncode.org/). DE genes are then identified by Student's *t*-test is performed to identify DE lncRNAs and mRNAs by calculating the fold change (FC) and *P*-value. Screening criteria for significant differences for upregulated and downregulated genes is FC > 2.0 and *P* < 0.05.

### 2.6. Gene Ontology (GO) and Kyoto Encyclopedia of Genes and Genomes (KEGG) Enrichment Analysis

Gene enrichment of the sequencing results of the DED disease model sequencing results can explore the most important biochemical metabolic and signal transduction pathways involved in the disease process. Gene Ontology (GO) and Kyoto Encyclopedia of Genes and Genomes (KEGG) data sets are used for pathway enrichment analysis. GO analysis of target genes is performed in the categories of biological process (BP), cellular component (CC), and molecular function (MF), while KEGG pathway analysis is applied to analyze the key regulatory pathways. The screening and mapping of differentially expressed genes are mainly accomplished via an online tool (https://cloud.oebiotech.cn).

### 2.7. CeRNA Network Analysis

The top 10 upregulate DE lncRNAs and DE mRNAs had a significant positive correlation (correlation coefficient >0.95) which are chosen as the target for the competing endogenous RNA analysis. MiRBase22 is used to predict the target miRNAs of lncRNAs from all known mouse miRNAs. The predicted target miRNAs acted as a bridge linking the lncRNAs and mRNAs to form the lncRNA-miRNA-mRNA network, which contains 96 links, drawn by Cytoscape.

### 2.8. Cell Culture and Transfection

The mouse corneal epithelial cell lines (MCECs) are purchased from ICell Bioscience Inc. (Shanghai, China). The cells are cultured in Dulbecco's Modified Eagle's Medium/Nutrient Mixture F12 Ham (DMEM/F12; Gibco, USA) containing 100 U/ml penicillin, 100 U/ml streptomycin (Gibco), 10% fetal bovine serum qualified Australia origin (FBS; Gibco, Catalog number:10099141, Australia), 1% non-essential amino acids (HyClone, USA), and 10 ng/ml mouse epithelial cell growth factor (PeproTech, USA). Cells are incubated in a humidified 37°C incubator containing 5% CO2.

siRNAs targeting NONMMUT047964.2 and the control siRNA are designed and synthesized by Getein Biotech lnc. (Jiangsu, China). When the cell confluence reached 70%, siRNAs are transfected into cells by using EndofectinTM MAX (GeneCopoeia, USA) according to the manufacturer's instructions. 24 hours after transfection, the culture medium is changed. When the cell confluence reached 80%, cell is treated with 450 mOsm/L culture medium which is prepared by using 90 mM sodium chloride. Cells are harvested by trizol for RT-qPCR after 24 hours of the above-mentioned treatment.

### 2.9. Annexin V/FITC Apoptosis Assay

After transfection and saline solution treatment, the cells are dissociated with trypsin into a 1.5 ml centrifuge tube. 3 × 105 cells are diluted with cell staining solution and then stained with 5 *μ*l Annexin V-FITC and 5 *μ*l PI at room temperature for 20 minutes. The samples are tested by the Cytoflex Flow Cytometer (Beckman, USA).

### 2.10. Real-Time qPCR

Total RNA is isolated from mouse cornea and MCECs by using Trizol reagent (Thermo). This experiment uses Nanodrop 2000 (Thermo) to control the quality of RNA. CDNA is synthesized using a fast miRNA Reverse Transcription Kit (ESscience, China) and a Fast All-in-One RT kit (ESscience, China). The RT-qPCR is run in a CFX Connect Real-Time System (Bio-RAD, USA) using SYBR green master mix (ESscience, China) and specific forward-reverse primers. The special primers used in the experiment could be referred to supplement file 1.

### 2.11. Statistical Analyses

Statistical analyses are performed using GraphPad Prism 5.0 (GraphPad Software, Inc., San Diego, CA, USA) software. Comparisons between groups are assessed using *e* paired *t*-test or the matched-pairs signed-rank test. *P* < 0.05 is considered statistically significant. Results are presented as mean ± standard deviations.

## 3. Results

### 3.1. DED in the Mouse Model

The 8-week-old c57bl/6 mice are placed in a dry and flowing environment and subcutaneously injected with scopolamine hydrobromide four times a day to construct the mice DED model. We conducted corneal fluorescein sodium staining and Schirmer's I-test at 0, 2, and 4 weeks, as shown in Figure 1(a). Before the treatment, we found no difference in fluorescence score and tear production between the two groups. The fluorescein scores at day 14 and day 28 after the injection significantly increased in the cornea of the DED mice compared to the control (8.33 ± 1.155 at 2 weeks, and 11.67 ± 0.577 at 4 weeks; *P* < 0.01, as shown in Figures 1(b) and 1(c). Moreover, tear production rapidly and significantly reduced at day 14 and day 28 (1.33 ± 0.29 mm/30 s at day 14, and 0.83 ± 0.29 mm/30 s at day 28; *P* < 0.05) in the DED compared with the control animals, as shown in Figures 1(d) and 1(e). After 28 days of subcutaneous injection, some of the mice's eyes were removed and stained with HE. The number of cell layers of corneal epithelium increased, the arrangement of cells in each layer is disordered, and the thickness of corneal epithelium increased in mixed dry eye mice, as shown in Figure 1(f).

### 3.2. Differential Expression of mRNAs, lncRNAs in DED Mouse

Based on the above fluorescence score and tear production results, the DED group is selected for the next ceRNA analysis. The expression profiles of mRNAs, lncRNA in DED mouse cornea are analyzed using microarray technology. A total of 289 mRNAs are identified to be upregulated and 411 mRNAs are downregulated. There are 856 DE lncRNAs, including 433 upregulated and 423 downregulated lncRNAs.  Figure 2(a) shows the DE lncRNA and Figure 2(b) shows mRNA that is ranked by FC, including both upregulated and downregulated. Volcano plot analysis is used to assess the variations in lncRNA, as shown in Figure 2(c).  Figure 2(d) shows mRNA's expression profiles between the DED group and control group.  Table 1 shows the top five most significant lncRNAs upregulated or downregulated in the DED group compared to the control. In order to verify the validity of the microarray analysis, we select 3 pairs of lncRNAs and 2 pairs of mRNAs for RT-qPCR verification, as shown in Figure 2(e). The results show that lncRNA NONMMUT047964.2 and NONMMUT054540.2 in DED are significantly increased compared with the control group, while the level of ENSMUST00000229379.1 expression is significantly reduced (*P* < 0.01). Then the between-group differences mRNAs Grm2 and Egr-1 are verified, revealing significantly upregulated, as shown in Figure 2(f).

### 3.3. GO and KEGG Analysis of the DE mRNAs

GO analysis results showed that changes in biological processes (BP) of DEGs are significantly enriched in negative regulation of angiogenesis, collagen fibril organization, pituitary gland development, response to virus, positive regulation of collagen biosynthetic process, positive regulation of mitochondrial fission, multicellular organism development, and embryonic limb morphogenesis, mesoderm formation, as shown in Figures 3(a) and 3(b). Changes in cell component (CC) of DEGs are mainly enriched in proteinaceous extracellular matrix, extracellular matrix, extracellular region, extracellular space, basement membrane, plasma membrane, presynaptic membrane, L-type voltage-gated calcium channel complex, voltage-gated calcium channel complex, and postsynaptic density. Changes in molecular function (MF) are mainly enriched in calcium ion binding, heparin binding, collagen binding, fibronectin binding, oxidoreductase activity, acting on paired donors, with incorporation or reduction of molecular oxygen, calcium-dependent phospholipase A2 activity, sulfotransferase activity, calcium channel activity, and extracellular matrix binding. Among the KEGG pathway analysis of upregulated mRNA, ether lipid metabolism signaling pathway is the most enriched, followed by proximal tubule bicarbonate reclamation and TGF-beta signaling pathway. Besides, GnRH signaling pathway, Ras signaling pathway, MAPK signaling pathway, TGF-beta signaling pathway, PI3K-Akt signaling pathway, and TNF signaling pathway, associated with inflammation, are also detected to be highly enriched, as shown in Figure 3(c).

### 3.4. CeRNA Network Analysis

Co-expressed lncRNAs and mRNAs are selected to predict the association with miRNAs. The top 10 upregulated lncRNAs and all the upregulated mRNAs are chosen to construct the ceRNA network, contained 96 relationship pairs, as shown in Figure 4. To verify the effectiveness of the constructed ceRNA network, two pairs of lncRNA-miRNA-mRNA pairs (NONMMUT047964.2-miR-671-5p-Egr-1 and NONMMUT 054540.2-miR-1934-5p-Grm2) are selected for validation at the cellular and tissue levels. First, we determined the level of miR-1934-5p and miR-671-5p expression in mouse corneal tissue samples.

In Figure 4, the red Diamond represent miRNAs, blue Square nodes represent mRNAs, and Cyan triangle nodes represent lncRNAs.  Figure 5, shows competing endogenous RNA interaction network of circRNA-miRNA-mRNA. Red represents upregulated expression, whereas green represents downregulated expression. Diamond nodes represent circRNAs, triangular nodes represent miRNAs, and oval nodes represent mRNAs. Hub genes are indicated by red boxes.circRNA, circular RNA; FC, fold change; miRNA/miR, microRNA (see this image and copyright information in PMC).

MiR-1934-5p and miR-671-5p are found to decrease significantly in the DED group compared with the control, in line with expected trends, as shown in Figure 5(a). Then, the cells are cultured under hypertonic conditions to simulate the hyperosmotic pressure in mice with dry eye disease. Similarly, we measured the mRNA expression levels of these pairs of relationships. The expression levels of NONMMUT047964.2, NONMMUT054540.2, Egr-1, and Grm2 are significantly increased and in MCECs after treated with 450 mOsm/L Culture medium. Meanwhile, the expression level of miR-1934-5p is found to be downregulated in the experimental group, as shown in Figure 5(b). The expression level of miR-671-5p is found to be downregulated in the experimental group, as shown in Figure 5(c). The results of qPCR indicated that co-expression existed in the tissues and cells of the two pairs selected, which proved the validity of ceRNA network.

### 3.5. Inhibition of NONMMUT047964.2 Expression Suppresses Cell Inflammation and Apoptosisure

The NONMMUT047964.2-miR-671-5p-Egr-1 axis is found to be differentially expressed in both corneal epitheliums of DED mice and MCECs treated with hypertonic culture medium. Early growth response 1 (Egr-1), the most significant gene upregulation in the microarray data, is seen as a positive modulate inflammatory gene. It mediates its effects by regulating the transcription of a wide array of downstream genes involved in inflammation, matrix formation, thrombosis, and apoptosis [9].We hypothesize that NONMMUT047964.2 may promote inflammation via the miR-671-5p/Egr-1 axis. To verify this hypothesis that NONMMUT047964.2 is involved in inflammatory insults, and siRNA-mediated knockdown experiments on the NONMMUT047964.2 are performed in MCECs by transfection. MCECs are divided into three groups: blank control group without any treatment, cells cultured under high osmotic pressure after transfection of negative double stranded siRNA, and cells cultured under high osmotic pressure after knockdown of NONMMUT047964.2. Validation of lncRNA NONMMUT047964.2 is shown in Figure 6.

## 4. Conclusion

In conclusion, our study constructed a model of mixed dry eye disease by exposure to a dry flowing environment and subcutaneously injected scopolamine, and first reported transcriptome sequencing analysis of mixed dry eye disease. We analyze ncRNA expression in the presence of decreased aqueous tear secretion reduction and constructed the network between lncRNA, miRNA, and mRNA. So far, the role of most lncrnas in dry eye is not fully understood. This study showed that there are 856 lncRNAs and 700 mRNAs differentially expressed in mixed dry eye mice. After transfection with siRNA of NONMMUT047964.2, IL-1*β* in MCECs is significantly decreased, and apoptosis rate is declined in hypertonic environment. In addition, we speculate that NONMMUT047964.2 may play an important role in the inflammatory process of DED through miR-671-5p/Egr-1. The results of this study may lead to a deeper understanding of the pathogenesis of mixed dry eye, and provide a potential regulatory mechanism of lncRNA in DED on inflammation and a potential new therapeutic target of lncRNA [18].

## Figures and Tables

**Figure 1:** Identification of DED in mouse model: (a) administration of subcutaneous injection of scopolamine for 4 weeks in DED group. Examinations were taken at week 0, week 2, and week 4; (b) representative images of fluorescein staining on week 0, week 2, and week 4 in mixed DED group compared with images of the controls; (c) the fluorescein staining score of DED mice's corneas were significant increasing during molding process at week 0, week 2 and week 4 (*P* < 0.01); (d) representative images of wetted cotton thread in mixed DED group compared with the controls (*P* < 0.05); (e) tear production of mice in DED group was significantly decreased after injection of scopolamine and was much smaller than that in control group during the whole modeling process; and (f) HE staining images of mouse corneal epithelium after model establishment. ^∗^*P* < 0.05, ^∗∗^*P* < 0.01, ^∗∗∗^*P* < 0.001. DED, dry eye disease.

**Figure 2:** . Bioinformatic analysis and qPCR verification of differentially expressed lncRNAs and mRNAs: (a) heatmap of expression levels of tissue-specific lncRNAs; (b) heatmap of expression levels of tissue-specific mRNAs; (c) volcano plot filtering identified 856 lncRNAs differentially expressed in DED group; (d) volcano plot filtering identified 700 mRNAs differentially expressed in DED group; (e) lncRNA NONMMUT047964.2, NONMMUT054540.2, ENSMUST00000229379.1 expression in DED and control mouse corneal tissues determined by qPCR analysis; and (f) the expression of Grm2 and Egr-1 in the tissue sample via RT-qPCR analysis. ^∗^*P* < 0.05, ^∗∗^*P* < 0.01, ^∗∗∗^*P* < 0.001. DED, dry eye disease.

**Figure 3:** GO and KEGG analysis of the DE mRNAs: (a) the barplot of top 30 enrichment pathway by upregulating DE mRNA by go analysis; (b) the bubble plot of top 30 enrichment pathway by upregulating DE mRNA by go analysis; and (c) the bubble plot of top 30 enrichment pathway by upregulating DE mRNA by KEGG analysis. GO, Gene Ontology. KEGG, Kyoto Encyclopedia of Genes and Genomes.

**Figure 4:** The ternary regulatory network of lncRNA-miRNA-mRNA.

**Figure 5:** Verification of ceRNA relation pairs: (a) the expression of miR-671-5p and miR-1934-5p in mouse cornea; (b) the expression of NONMMUT054540.2, miR-1934-5p, and Grm-2 in hypertonic MCECs compared with control group; and (c) the expression of NONMMUT047964.2, miR-671-5p, and Egr-1 in hypertonic MCECs compared with control group.

**Figure 6:** Validation of lncRNA NONMMUT047964.2, regulating the inflammation and apoptosis in vivo: (a) flow cytometric analysis of MCECs apoptosis after treatment; (b) barplot of apoptosis after treatment; (c) the expression of IL-1*β*; (d) the expression of IL-6; (e) the expression of NONMMUT047964.2; (f) the expression of miR-671-5p; and (g) the expression of Egr-1 in MCECs following NaCl treatment.

**Table 1:** Top 5 upregulate and top 5 downregulate genes.

GeneID	log2FoldChange	Regulation	Chromosome	Control mean	DEDmean	*P*-value
NONMMUT111608.1	-3.280763851	Down	chr3	9.107995671	5.82723182	0.003616607
NONMMUT143900.1	-3.226411519	Down	chr15	5.638450123	2.412038604	0.023032577
ENSMUST00000229379.1	-3.127480369	Down	chr16	4.98460699	1.857126621	1.16E-05
NONMMUT083475.1	-3.102795346	Down	chr11	4.787754559	1.684959212	0.006322078
ENSMUST00000130262.1	-2.880416935	Down	chr2	5.691928277	2.811511342	0.000233881
NONMMUT047964.2	2.720766811	Up	chr4	1.219371013	3.940137824	0.000135135
NONMMUT100650.1	2.643541013	Up	chr17	1.140981357	3.784522369	5.28E-05
NONMMUT140691.1	2.534413029	Up	chr11	1.645556143	4.179969172	0.008430906
NONMMUT108663.1	2.518686891	Up	chr2	1.998732221	4.517419113	0.049224893
NONMMUT054540.2	2.461933599	Up	chr5	1.854416609	4.316350208	0.029071629

## Data Availability

The simulation experiment data used to support the findings of this study are available from the corresponding author upon request.
